The article "Gastroprotection Studies of Schiff Base Zinc (II) Derivative Complex against Acute Superficial Hemorrhagic Mucosal Lesions in Rats" was retracted in 2026. Reasons: duplicated data; overlap with earlier publications; unreliable results or conclusions; concerns about the data.

# Gastroprotection Studies of Schiff Base Zinc (II) Derivative Complex against Acute Superficial Hemorrhagic Mucosal Lesions in Rats

**DOI:** 10.1371/journal.pone.0075036

**Published:** 2013-09-13

**Authors:** Shahram Golbabapour, Nura Suleiman Gwaram, Pouya Hassandarvish, Maryam Hajrezaie, Behnam Kamalidehghan, Mahmood Ameen Abdulla, Hapipah Mohd Ali, A. Hamid A Hadi, Nazia Abdul Majid

**Affiliations:** 1 Department of Biomedical Science, Faculty of Medicine, University of Malaya, Kuala Lumpur, Malaysia; 2 Department of Chemistry, University of Malaya, Kuala Lumpur, Malaysia; 3 Institute of Biological Science, Faculty of Science, University of Malaya, Kuala Lumpur, Malaysia; 4 Department of Pharmacy, Faculty of Medicine, University of Malaya, Kuala Lumpur, Malaysia; Center for Cancer Research, National Cancer Institute, United States of America

## Abstract

**Background:**

The study was carried out to assess the gastroprotective effect of the zinc (II) complex against ethanol-induced acute hemorrhagic lesions in rats.

**Methodology/Principal Finding:**

The animals received their respective pre-treatments dissolved in tween 20 (5% v/v), orally. Ethanol (95% v/v) was orally administrated to induce superficial hemorrhagic mucosal lesions. Omeprazole (5.790×10^−5^ M/kg) was used as a reference medicine. The pre-treatment with the zinc (II) complex (2.181×10^−5^ and 4.362×10^−5^ M/kg) protected the gastric mucosa similar to the reference control. They significantly increased the activity levels of nitric oxide, catalase, superoxide dismutase, glutathione and prostaglandin E2, and decreased the level of malondialdehyde. The histology assessments confirmed the protection through remarkable reduction of mucosal lesions and increased the production of gastric mucosa. Immunohistochemistry and western blot analysis indicated that the complex might induced Hsp70 up-regulation and Bax down-regulation. The complex moderately increased the gastroprotectiveness in fine fettle. The acute toxicity approved the non-toxic characteristic of the complex (<87.241×10^−5^ M/kg).

**Conclusion/Significance:**

The gastroprotective effect of the zinc (II) complex was mainly through its antioxidant activity, enzymatic stimulation of prostaglandins E2, and up-regulation of Hsp70. The gastric wall mucus was also a remarkable protective mechanism.

## Introduction

Zinc, the second most abundant transition metal, is an essential trace element with a variety of biological roles in organisms [1]–[3]. It stabilizes macromolecules [4] and is critical in storage routines, transcription factors, and replication proteins [5], [6]. Involved in various metabolisms of genome [7]–[10] and proteins [11]–[13], zinc is a vital biological element (for a review, see [14]). Variation in structural configuration of zinc proteins introduced zinc as the only metal which appears in all six fundamental enzyme classes; oxidoreductases, lyases, hydrolases, transferases, ligases, and isomerases [15]. Zn^2+^ possesses lewis acid properties [16] and redox activity [17]. Zinc based compounds potentially may have a variety of therapeutic activities which makes it an attractive element in drug therapy. Analogous zinc compound has anti-bacterial activity against gram-positive bacteria [1]. Zinc controls bacterial gene expression for instance, bacterial proteins such as the iron responsive regulator fur, alcohol dehydrogenases, hydrolases, lyases, and Cu/Zn superoxide dismutases utilize zinc [18]–[20]. The effectiveness of the zinc (II) complex in preventing mucosal damage might inhibit pathogenesis activity of bacteria in the gastrointestinal (GI) tract.

Inflammatory reactions are governed by histamine, bradykinin, serotonin, prostaglandins, the blood clotting system, and T cells (lymphokines) [21]. Essential for T-cell proliferation, activation of extracellular signal regulated kinase 2 in response to IL-2 is dependent on zinc [21]. Zinc signals in neutrophil granulocytes are required for the formation of neutrophil extracellular traps [22]. The presence of bromine atoms coordinated to the zinc metal ion seemed a possible active site for the complex and this might be ascribed to the electron donating properties of the halogens by resonance, making the lone pair electrons more available to a plausible electron transfer (for a review, see [23], [24]). Similarly, bromine substituted copper complex showed amazing gastroprotective activity [25]. Analogous zinc coordinated Schiff base compounds demonstrated potential urease inhibition [26]–[28]. This mechanism might be performed by this complex as a potential treatment for eradicate *helicobacter pylori* and prevent further recurrence of ulcer after therapy. Studies showed that antioxidant activity is important in gastroprotection. Several natural/synthetic agents introduced with protective effects against acute hemorrhagic gastric lesions possessed free-radical scavenging activity [29]–[33]. The antioxidant activity of several ingredients might augment the total antioxidant activity of the tissue [30], [34]. Another protective mechanism is the suppression of acid secretion which have been considered a preventive strategy against gastric superficial hemorrhagic mucosal lesions. For instance, proton pump inhibitors (PPIs) are effective agents in inhibiting gastric acid secretion [35]. Previous studies on Zn (II) [benzenesulfanohydrazide] [36] and Zn (II) [piperazine] [37] showed remarkable gastroprotection. In this study, synthesized Schiff base zinc (II){Dichlorido-2-morpholino-*N*-[1-(2-pyridyl)ethylidene] ethanamine *k^3^ N,N’,N”}* was evaluated for its gastroprotective activity against acute hemorrhagic gastric mucosal lesions in normal rats.

## Materials and Methods

### Synthesis of the Complex

In this study, the chemicals were obtained from Fluka and Aldrich, and used without further purification. Zinc (II) complex (Figure 1) was synthesized by condensation reaction of 2-acetylpyridine and 4-(2-aminoethyl)morpholine followed by complexation of the ligand with zinc (II) acetate dihydrate in the presence of potassium bromide [38]. Briefly, the product was collected by filtration, washed several times with ethanol until a milky coloured precipitate was obtained. The precipitate was dried in a vacuum desiccator. Recrystallization was performed in a mixture of methanol and dichloromethane. The x-ray crystal structure of the zinc (II) complex was previously published [39]. Infrared spectra were obtained using KBr discs (4000–400 cm^−1^) on Perkin –Elmer FT-IR spectrometer. ^1^H and ^13^C NMR spectra were recorded on Jeol JNM-LA400 FT-NMR system (Figures S1 and S2). TMS was used as an internal standard and deuteriated DMSO-*d6* as a solvent. Elemental analysis (C, H, N) were performed using a Flash EA 1112 Series elemental analyser in the University of Technology Malaysia. Elemental analysis and spectral characterization for the ligand and its metal complex was previously published by Gwaram *et al.* [38].

**Figure 1:** Chemical structure of the zinc (II) complex [38].

### Animals

*Sprague Dawley* and ICR mice rats were attained from Animal House, Faculty of Medicine, University of Malaya, Kuala Lumpur. The animals were housed in an isolated cabin maintained at ∼24°C in a relative humidity of 80% using an automated ventilation system. An artificial lighting system was used for a daily ratio of 1∶1. Animals had access to standard rat pellets and tap water *ad libitum*. In our preliminary study (unpublished data) and on the basis of acute toxicity results, different doses of the zinc (II) complex were examined in rats to find effective doses for gastroprotection.

### Ethical Issues

All procedures were performed in compliance with the National Institutes of Health Guide for the care and use of Laboratory Animals [40] and approved by the committee for animal experimentation- Faculty of Medicine, University of Malaya [University of Malaya- Ethic No. (ISB/30/05/2012/SG (R)]. Throughout the experiments, all of the animals received humane care according to the “Guide for the Care and Use of Laboratory Animals” prepared by the National Academy of Sciences [41].

### Drugs and Chemicals

In this study, a dilution (5% v/v) of tween 20 (Merck, Germany) was used as the vehicle. Omeprazole, the reference drug for prevention of superficial hemorrhagic mucosal lesions, was obtained from UMMC and dissolved in the vehicle (5% tween 20).

#### Toxicity evaluation

The acute toxicity study was performed in accordance with the OECD protocol [40]. The acute toxicity study was to determine a non-toxic range of doses for the zinc (II) complex. Thirty six mice (18 males and 18 females, 6–8 weeks old) were assigned randomly into three groups (for each gender) and were administrated orally with the vehicle (5% tween 20), 43.621×10^−5^ M/kg or 87.241×10^−5^ M/kg of the zinc (II) complex (5% tween 20), accordingly. Prior to the dosing, the animals were fasted for 24 h (water was accessible but the last 2 h). Water and food was suspended for another 1 and 3 h after dosing, respectively. During the first 48 h, animals were monitored for any sign of abnormality. Onwards, they were examined for their health condition, twice per day. The Animals were under assessment for a period of 14-day to record any sign of toxicity or mortality. The animals were euthanized on day 15 for histology and hematology evaluations.

### Ethanol-induced Lesion

Preventive effect of the zinc (II) complex against superficial hemorrhagic mucosal lesions were assessed in the normal rats. 48 rats were randomly divided into 8 groups of 6 individuals; the normal control group, the complex control group (8.724×10^−5^ M/kg of the zinc (II) complex), the lesion control group, the reference control group (5.790×10^−5^ M/kg omeprazole) and 4 experimental groups (1.091×10^−5^, 2.181×10^−5^, 4.362×10^−5^ and 8.724×10^−5^ M/kg of the zinc (II) complex). Table 1 shows specifications for each group. The vehicle was orally administrated (5 mL/kg) to the normal control and the lesion control as a pre-treatment. The vehicle also was given orally to the normal control and complex control groups as a treatment. A single treatment with ethanol (95% v/v), was orally (5 mL/kg) administrated to the lesion control group, reference control group and the experimental groups. Prior to the pre-treatment, the rats were fasted for 24 h (water was accessible but the last 2 h). The interval between the pre-treatment and the treatment was 60 min. The animals were euthanized 60 min after the treatment with an over-dose of xylazine and ketamine anesthesia and their stomachs were immediately excised.

**Table 1:** The experimental design and specifications.

Groups	Description	Pre-treatment	Treatment
**Group 1**	Normal control	5% tween 20	5% tween 20
**Group 2**	Complex control	Complex 8.724×10^−5^ M/kg	5% tween 20
**Group 3**	Lesion control	5% tween 20	95% ethanol
**Group 4**	Reference control	omeprazole 5.790×10^−5^ M/kg	95% ethanol
**Group 5**	Experimental group1	Complex 1.091×10^−5^ M/kg	95% ethanol
**Group 6**	Experimental group 2	Complex 2.181×10^−5^ M/kg	95% ethanol
**Group 7**	Experimental group 3	Complex 4.362×10^−5^ M/kg	95% ethanol
**Group 8**	Experimental group 4	Complex 8.724×10^−5^ M/kg	95% ethanol

### Macroscopic Appearance of Lesions

Acute hemorrhagic gastric lesions were characterized grossly. In accordance with several studies, the superficial mucosal lesions were petechial and hemorrhagic in different bund sizes, parallel to the long axis of the stomach [25], [31], [33], [37], [42], [43]. Luminal surface of each stomach was assessed for the hemorrhagic damage. To calculate the protection percentage (P%) for each pre-treatment, the lesion area (LA) was calculated using a dissecting microscope (1.8×) and a planimeter (10×10 mm^2^) where LE and LG were lesion area of the lesion control and lesion area of a given group, respectively.


### Evaluation of Mucosal Protective Factors

Previous studies showed that several gastroprotective mechanisms were involved in the protection of gastric tissue against aggressive conditions [25], [30], [34]. The acidity of gastric juice, gastric wall mucosa, antioxidant and enzymatic activities of the stomach were assessed to identify protective mechanisms of zinc (II) complex in the ethanol-induced gastric lesions in rats.

#### Measurement of gastric juice acid content

In order to measure the acidity of gastric juice, after dissecting the stomach, its contents drained into a falcon tubes and centrifuged at 4000 rpm for 10 min. The supernatant pH was recorded with a digital pH meter.

#### Gastric mucus production

Gastric wall mucus production was measured for each group [44]. Briefly, after removing the glandular segments, the stomach tissue was immersed in 1% Alcian blue solution (in sucrose solution, buffered with sodium acetate at pH 5) and was rinsed with sucrose solution to remove the excess dye. Magnesium chloride solution (500 mM) extracted the dye from the mucus-dye complex. The extract mixed with diethyl ether was centrifuged at 3000 rpm for 10 min and the absorbance of supernatant was measured at 580 nm to calculate the content of alcian blue extracted (µg of alcian Blue) per gram of glandular tissue.

#### Enzymatic activities of stomach tissue homogenate

For each rat, the gastric tissue homogenate was prepared in phosphate-buffered saline (PBS) at ∼4°C (125 mg tissue/mL PBS). The tissues were homogenized with a teflon homogenizer (Polytron, Germany). After centrifugation at 4,500 rpm for 15 min at 4°C, the supernatant was used for the enzymatic and protein assays.

#### Antioxidant activities and formation of prostaglandins E2 of stomach homogenate

The nitric oxide (NO), catalase (CAT), glutathione (GSH) and superoxide dismutase (SOD) levels of the gastric tissues were measured using commercial kits (Cayman, USA). The gastric tissue supernatant of each sample was subjected to the assays according to the manufacturer protocols. The levels of prostaglandin E2 (PGE-2) and malondialdehyde (MDA) in the gastric tissue supernatant were measured using commercial kits (Cayman, USA). Protein concentrations were determined through Biuret reaction [45].

### Histological Analysis

Specimens of the gastric tissue were fixed using 10% buffered formalin, were processed in the paraffin tissue-processing machine (Leica, Germany), and were embedded in paraffin blocks. Sections of 5 µm were subjected to hematoxylin and eosin (H&E) staining and periodic acid schiff (PAS) staining (Sigma Aldrich, Malaysia). H&E staining was to evaluate the tissue architecture. Periodic acid schiff (PAS) staining was to evaluate changes in glycoproteins (acidic and basic) and to observe the produced mucus. The gastric sections were observed and photographed under a light microscope (Nikon, Japan).

### Immunohistochemistry Analysis

Specimens of the gastric tissue were fixed (10% buffered formalin) and processed in the paraffin tissue-processing machine (Leica, Germany). Sections of 5 µm were placed on 3-aminopropyltrimethoxysilane (APES)-treated glass slides and were subjected to the immunochemical staining Hsp70 (Abcam, USA) and Bax (Abcam, USA), using a streptavidin peroxidase (Abcam, USA).

### Western Blot Analysis

For western blot analysis, proteins were extracted from the same gastric mucosa samples using protein extraction buffer (Pierce, USA), the gastric tissue supernatant of each sample was subjected to the western blot assays according to the previously published procedure [46], [47], with some modifications. Proteins (30 µg) were separated by 12% SDS-PAGE (25 mA, for 2 h). Proteins were transferred to PVDF membranes (Pierce, USA) using a Trans-Blot SD semi-dry transfer cell (Bio-Rad, USA) at 15 V, 95 mA, for 1 h. The PVDF membrane was blocked using Blocker™ Casein (Pierce, USA) for 1 h at room temperature and washed twice using TBST. The membranes were then incubated at 4°C overnight with primary antibodies; Hsp70 mouse monoclonal antibody (1∶1000; Santa Cruz Biotechnology, USA), Bax mouse monoclonal antibody (1∶1000; Santa Cruz Biotechnology, USA) and β-actin mouse monoclonal antibody (1∶1000; Santa Cruz Biotechnology, USA). The membranes were then incubated for 1 h at room temperature with goat anti-mouse and goat anti-rabbit secondary antibodies conjugated with alkaline phosphatase (i-DNA, USA) at a ratio of 1∶1000, then washed twice with TBST for 10 min. The blotting were developed using the BCIP/NBT (Santa Cruz Biotechnology, USA) solution for a period of 5–30 min to detect the target protein band as a precipitated dark blue colour.

### Statistical Analysis

The data was analysed using analysis of variance by ANOVA analysis followed by post-hoc analysis. A value of *p<*0.05 was considered significant. The data was analysed using the IBM SPSS version 20 (IBM Corporation, USA) statistical software [48]. The data is expressed as means ± standard error.

## Results

### Acute Toxicity Study

For duration of 14 days, none of the individuals in the acute toxicity test showed any sign of abnormality or toxicity. Histological assessment did not show any sign of nephrotoxicity and/or hepatotoxicity. Hematological and serum biochemical parameters were reported normal (Figure S3 and Table S1). The lethal dose, 50% (LD_50_) for male and female mice were 1352.23 M/kg and 1169.02M/kg, respectively.

### Macroscopic Evaluation of Gastric Lesions

As a pre-treatment, four doses of the zinc (II) complex (1.091×10^−5^, 2.181×10^−5^, 4.362×10^−5^ and 8.724×10^−5^ M/kg) were examined against the ethanol-induced gastric lesions in the normal rats. Macroscopic evaluation of the lesions and the comparisons among different groups showed that the doses of 1.091×10^−5^ M/kg and 2.181×10^−5^ M/kg of the zinc (II) complex had the most remarkable protective effects (*p*<0.05) after the reference group (5.790×10^−5^ M/kg omeprazole). Table 2 presents the inhibition percentage among the groups. Ethanol caused extensive and remarkable hemorrhagic lesions on the gastric epithelium. The pre-treatment with the omeprazole or the zinc (II) complex significantly protected the gastric mucosa against the damage (Table 2).

**Table 2:** Measurement of the lesion area, inhibition percentage, alcian blue binding capacity and pH.

Groups	Ulcer area (mm)^2^	Inhibition	pH	GWM
**Group 1**	0* ^#^ ±0	0	4.60* ^#^ ±0.02	696.23* ^#^ ±3.41
**Group 2**	0* ^#^ ±0	0	4.70* ^#^ ±0.02	716.59* ^#^ ±1.54
**Group 3**	970.13# ±21.12	0	3.71* ^#^ ±0.03	117.30# ±5.12
**Group 4**	124.60* ±5.38	87%	5.95* ^#^ ±0.06	613.77* ±6.66
**Group 5**	201.10* ^#^ ±8.16	79%	4.19* ^#^ ±0.03	552.16* ^#^ ±6.13
**Group 6**	136.92* ±7.41	86%	5.22* ^#^ ±0.04	588.51* ^#^ ±4.51
**Group 7**	159.06* ±2.79	84%	5.38* ^#^ ±0.09	570.35* ^#^ ±4.35
**Group 8**	200.62* ^#^ ±5.19	79%	5.52* ^#^ ±0.06	546.74* ^#^ ±7.18

The experiment consisted of the negative control group (Group 1), the complex control group (Group 2), the lesion control group (Group 3), the reference group pre-treated with 20 of omeprazole (Group 4) and the experimental groups (Groups 5–8) which received 1.091×10^−5^, 2.181×10^−5^, 4.362×10^−5^ and 8.724×10^−5^ M/kg of the zinc (II) complex as a pre-treatment. All values are expressed as mean ± standard error mean. Mean difference is significant at the *p*<0.05 level (one-way between groups ANOVA with post-hoc analysis).

* significant when compared to the ulcer control group (Group 3).

# significant when compared to the reference control group (Group 4).

### Evaluation of Mucosal Protective Factors

#### Measurement of gastric juice acid content (pH)

Table 2 represents the acidity of the gastric juice of the rats. The highest pH was recorded in the reference control group (p<0.05).

#### Gastric mucus production

Alcian-blue-binding capacity for each group was compared with the lesion control group (Group 3) and the reference control group (Group 4). Table 2 shows the differences in the capacity for each group. The normal control group and the complex control group showed a similar binding capacity (p<0.05). In comparison, the lesion control group possessed the lowest capacity. The pre-treatment with the omeprazole or with the complex in the experimental groups significantly compensated the lost capacity imposed by ethanol. Among the experimental groups, the pre-treatment with 2.181×10^−5^ M/kg and 4.362×10^−5^ M/kg were relatively the highest and close to that of the reference control group.

#### Protein concentration

Protein concentration for the complex control group was the highest and the reference control group showed non-significant differences to the experimental groups but Group 5 (Table 3).

**Table 3:** Measurement of the total protein concentration, antioxidant activity, lipid peroxidation and formation of prostaglandins E2 of the tissue homogenates.

Groups	Protein (mg/ml tissue)	NO (µM)	CAT nM/min/ml	SOD (U/mg protein)	GSH (µM/mg protein)	MDA (µM/g protein)	PGE-2 (ng/mg protein)
**Group 1**	14.72* ^#^ ±0.23	9.15* ^#^ ±0.08	125.88* ^#^ ±3.43	15.96* ^#^ ±0.41	16.81* ^#^ ±0.20	99.41* ^#^ ±3.63	3.56* ^#^ ±0.03
**Group 2**	15.53* ^#^ ±0.39	8.79* ^#^ ±0.14	129.35* ^#^ ±1.03	16.40* ^#^ ±0.19	17.32* ^#^ ±0.17	87.14* ^#^ ±4.71	3.65* ^#^ ±0.02
**Group 3**	9.18# ±0.23	3.64# ±0.11	66.56* ^#^ ±2.33	11.42# ±0.29	9.87# ±0.39	206.43# ±3.48	1.16# ±0.006
**Group 4**	13.39* ±0.15	7.99* ±0.19	151.79* ^#^ ±4.39	27.43* ±0.26	14.49* ±0.18	128.80* ±5.11	3.29* ±0.02
**Group 5**	11.99* ^#^ ±0.26	5.33* ^#^ ±0.05	145.30* ±1.28	19.56* ^#^ ±0.19	11.13* ^#^ ±0.20	101.59* ^#^ ±3.68	2.18* ^#^ ±0.006
**Group 6**	12.67* ±0.41	7.19* ^#^ ±0.08	149.56* ±0.80	26.77* ±0.12	14.21* ±0.48	99.24* ^#^ ±3.64	3.28* ±0.014
**Group 7**	13.50* ±0.31	6.90* ^#^ ±0.09	140.86* ^#^ ±0.77	25.30* ^#^ ±0.38	13.11* ^#^ ±0.19	127.72* ±6.00	3.26* ±0.002
**Group 8**	13.21* ±0.19	6.12* ^#^ ±0.09	142.13* ±0.94	24.96* ^#^ ±0.57	11.43* ^#^ ±0.26	113.30* ±3.98	3.15* ^#^ ±0.005

This experiment consists of the negative control group (Group 1), the complex control group (Group 2), the lesion control group (Group 3), the reference group pre-treated with 5.790×10^−5^ M/kg of omeprazole (Group 4) and the experimental groups (Groups 5–8) which received 1.091×10^−5^, 2.181×10^−5^, 4.362×10^−5^ and 8.724×10^−5^ M/kg of the zinc (II) complex as a pre-treatment. All values are expressed as mean ± standard error mean. Mean difference is significant at the *p*<0.05 level (one-way between groups ANOVA with post-hoc analysis).

* significant when compared to the ulcer control group (Group 3).

# significant when compared to the reference control group (Group 4). NO, nitric oxide; CAT, catalase; SOD, superoxide dismutase; GSH, glutathione; MDA, Malondialdehyde; PGE-2, prostaglandins E2.

#### Antioxidant activities and formation of prostaglandins E2 of stomach homogenate

Table 3 shows antioxidant and enzymatic activities of stomach tissue homogenates of the groups. The lesion control group showed a major reduction of the level of each antioxidant component (NO, CAT, GSH and SOD). In contrast, the pre-treatment with either the omeprazole or the complex in majority of the antioxidant assays compensated those reductions to maintained the levels. The pre-treatment with 2.181×10^−5^, 4.362×10^−5^ and 8.724×10^−5^ M/kg of the zinc (II) complex showed high level of activity for NO, but the reference control group showed the highest activity. The activity of CAT was significant in the rats pre-treated with the omeprazole (5.790×10^−5^ M/kg) or with the zinc (II) complex (1.091×10^−5^ and 2.181×10^−5^ M/kg). The levels of SOD and GSH in those rats pre-treated with omeprazole (5.790×10^−5^ M/kg) or the complex (4.362×10^−5^ M/kg) were significantly high. The normal control group and the complex control group did not show notable differences in the antioxidant assays.

The level of PGE-2 in the normal control group and the complex control group appeared the highest level among the groups. While the lesion control group showed the minimum formation of PGE-2, the pre-treatment with omeprazole (5.790×10^−5^ M/kg) or the complex (2.181×10^−5^ and 4.362×10^−5^ M/kg) recompensed the activity level, significantly. The lesion control group showed increase in the tissue level of MDA accompanied by impairment of anti-oxidative defence mechanisms. Unsurprisingly, the MDA levels were well maintained in the pre-treatment with either omeprazole (5.790×10^−5^ M/kg) or the zinc (II) complex (especially doses of 2.181×10^−5^ M/kg and 4.362×10^−5^ M/kg) in comparison to that of the lesion control group.

### Histological Evaluation

In compliance with the macroscopic appearance, histological evaluation of the gastric tissues showed different microscopic features as shown in Figure 2. An extensive superficial damage induced by ethanol was observed in the gastric mucosa of the lesion control groups. They showed extensive edema and leukocyte infiltration of the submucosal layer (Figure 2C). Histological examination indicated that the oral pre-treatment with omeprazole (5.790×10^−5^ M/kg) prevented the gastric tissue from hemorrhagic lesions (Figure 2D). Similarly, the pre-treatment with the zinc (II) complex showed the reduction of the lesion area, submucosal edema and leukocyte infiltration (Figures 2E–2H).

**Figure 2:** Hematoxylin and eosin staining evaluation of the gastric mucosa. The negative control and the complex control group have not any disruption to the gastric epithelium, submucosal edema or leucocyte infiltration (A). The lesion control group has extensive edema in the submucosal layer (B). Moreover acute hemorrhagic gastric lesions with severe disruption to the epithelium penetrated deeply into the mucosa (C) along with leucocyte infiltration are also noticeable (D and E). The pre-treatments with the complex (4.362×10^−5^ M/kg) show mild superficial disruption to the gastric epithelium (F).

The PAS staining was performed to assess the production of glycogen in the gastric epithelium. The gastric mucosa in the rats pre-treated with omeprazole (5.790×10^−5^ M/kg) or the complex (Groups 4–8) showed increase in PAS staining intensity comparing with the lesion control group in which the PAS staining not profusely noticeable. The glycoprotein content of gastric mucosa appeared almost similar in all groups but the lesion control group. Figure 3A shows the PAS staining of the gastric tissue received 4.362×10^−5^ M/kg of the complex.

**Figure 3:** Glycoprotein-PAS staining and immunohistochemical evaluation for the expression of Hsp70 and Bax proteins of the gastric mucosa. Oral administration of the zinc (II) complex (2.181×10^−5^ M/kg) increased the glycoprotein content of the gastric tissue (A), enhanced the expression of Hsp70 protein (B) and suppress the expression of Bax protein (C). The arrows point to the respective protein accumulations.

### Immunohistochemistry Evaluation

Immunohistochemical evaluation of the gastric tissues showed up-regulation of Hsp70 protein in gastric mucosa in the rats pre-treated with omeprazole (5.790×10^−5^ M/kg) or the complex- especially in the dose of 4.362×10^−5^ M/kg (Figure 3B)- when compared with the lesion control group. The normal control group and the complex control group also showed more expression of Hsp70 in comparison to the lesion control group. Immunohistochemical staining of Bax protein of gastric mucosa showed down-regulation of Bax protein in those groups pre-treated with the omeprazole (5.790×10^−5^ M/kg) or 4.362×10^−5^ M/kg of the zinc (II) complex (Figure 3C) while the lesion control groups showed up-regulation of the protein. In the normal control group, the immunohistochemistry of Hsp70 and Bax proteins was similar to the complex control group. Figure 3 (B and C) shows immunohistochemistry for the expression of Hsp70 and Bax proteins of the gastric tissues in the rat received 4.362×10^−5^ M/kg of the complex.

### Western Blot Assay

Western blot analysis confirmed the immunohistochemistry results. The complex (2.181×10^−5^ and 4.362×10^−5^ M/kg) and omeprazole (5.790×10^−5^ M/kg) caused up-regulation of Hsp70 protein in the pre-treated rats when compared with the normal control group (Figure 4A). The complex control group by itself caused mild up-regulation of the expression of Hsp70. In the lesion control group, the expression of this protein was remarkably down-regulated as compared with the normal control group (Figure 4A).

**Figure 4:** Western blot analysis with Hsp70 and Bax mouse monoclonal antibody. Corresponding β-actin blots are shown as a control for sample loading. G1, normal control; G2, complex control; G3, lesion control; G4, reference control; G5, zinc (II) complex (2.181×10^−5^ M/kg); G6, zinc (II) complex (4.362×10^−5^ M/kg).

The expression of Bax protein showed that the protein was up-regulated in the lesion control group as a strong sign of apoptosis while those rats pre-treated with omeprazole (5.790×10^−5^ M/kg) or the complex showed remarkable down-regulation of the expression of Bax protein (Figure 4A).

## Discussion

In recent years, the awareness of the implications of cyclooxygenase 2 on prevention and maintenance of gastric mucosal integrity and ulcer healing [49], [50] persuade several studies to find alternative therapeutics for preventing and treating superficial hemorrhagic mucosal lesions. Several studies have promoted ethanol-induced model of hemorrhagic gastric lesions [34], [51]–[53]. It has been established that one of the most important detrimental effects evoked by ethanol-induced gastric lesion is represented by increments of gastric mucosal MDA levels, a marker for oxidative stress [54]. ROS such as superoxide anions, hydrogen peroxide, and hydroxyl radicals, is the main cause of oxidation of biological constituents in gastric mucosal injury [55]. Ethanol, a necrotizing agent, induces cell membrane injury through generating free radicals [56]–[58] and lipid peroxidation [59], [60]. Increase in the permeability of the cell membrane causes extensive tissue destruction [61] which macroscopically appears as hemorrhagic erosions in the gastric mucosa. Moreover, oral administration of ethanol imposes vascular permeability and, diffuse severe damage to the capillaries of the gastric glandular mucosa [62] which in turn appears as petechiation or hemorrhagic bundles. Results of the several works demonstrated that, the effect of oral administration of ethanol on gastric functions was to reduce the gastric mucin content [31], [34], [37]. In the current study, the acute toxicity test did not show any sign of toxicity or mortality in the given dosages. In this study omeprazole was used as a reference medicine in prevention of gastric lesion. The idea was to compare the preventive activity of the zinc (II){Dichlorido-2-morpholino-*N*-[1-(2-pyridyl)ethylidene] ethanamine *k^3^ N,N’,N”}* complex with that of the reference medicine, omeprazole, in ethanol-induced gastric lesion rats. Omeprazole protected gastric mucosa significantly against the induced aggressive factor, ethanol. Omeprazole, a substituted benzimidazole derivative, is a proton pump inhibitor that inhibits gastric acid secretion [63] and managing acute hemorrhagic mucosal lesions. PPIs with antioxidant properties [64] inhibit acid secretion, and promote gastric epithelial cell migration [65]. However, its stimulating effect on mucus secretion has remained controversy [66]. In addition to the effectiveness of omeprazole on acid-dependent gastric lesion, it is also effective on acid-independent gastric model [67]–[70]. Ethanol, as it was shown in this study, causes severe macroscopic lesion with histological changes such as extensive edema, leukocyte infiltration of the submucosal layer and loss of integrity of gastroepithelium along with the impairment of gastric mucosa [30], [42]. In accordance with previous studies, our result showed that omeprazole (5.790×10^−5^ M/kg) prevented the reduction of protein concentration along with increase in PGE-2 [25], [30], [34]. In addition to a newly published research on anti-ulcer effect of a synthesized steroid [34], our study provided an evidence on gastroprotective effect for PG through increasing the formation of PGE-2 [71].

The zinc (II) complex (as shown in the complex control group) not only maintained the normal condition of the stomach but to some extents enhanced the defensive efficacy of the tissue. The antioxidant activity of the pre-treatment with the zinc (II) complex was increased in the gastric homogenates similar to the antioxidant activities of the reference medicine [72]. This study in consistence with several studies showed that antioxidant property was one of the main gastroprotective mechanisms [29], [33], [42], [53]. The Zn (II) complex appeared effective in the mid doses (2.181×10^−5^ and 4.362×10^−5^ M/kg). The highest dose (8.724×10^−5^ M/kg) appeared comparatively less effective in the protection against acute gastric lesions. Perhaps the main reason for such negative protective feedback lied in pro-oxidant activity of the Zn (II) complex in higher concentrations. Previous studies indicated that some Schiff base compounds might possess pro-oxidant property [73]–[76], however, a precise project should be conducted to show the exact pro-oxidation activity of the Schiff base Zinc (II) derivative complex.

The macroscopic and microscopic assessment among the reference group and the pre-treated rats with the zinc (II) complex (Groups 5–8) showed remarkable protection of gastric epithelium from ethanol-induced hemorrhagic lesion in a similar pattern to the reference control group. Consistent with previous studies [25], [34], [37], the gastric mucosal content increased remarkably in those groups that were pre-treated with the complex (Group 5–8), when compared to the lesion control. In comparison with the lesion control group, the reference control group among all the groups showed the highest level of the mucus content, but significant boost in mucosal content of Groups 5–8 (pre-treated with the complex) was noticeable. The zinc (II) complex enhanced the gastric mucosal content in the complex control group when compared with the normal control. These findings showed that the complex had the ability to stimuli the mucus secretion. In agreement with several studies [33], [34], [69], [70], [77], our investigation revealed that the exposure of gastric mucosa to oxidative stress was restricted through the oral administration of omeprazole (5.790×10^−5^ M/kg) or the complex as a pre-treatment. The involvement of formation of PGE-2 in the gastroprotective mechanisms was previously investigated with conflicting evidences [25], [29], [33], [34]. PGE-2, the most abundant GI prostaglandin, is fundamentally important in the regulation of gastric mucus secretion [78], gastric acid secretion [79] and gastric motility [80], [81]. In oral administration of ethanol, reduction in formation of PGE-2 lessened acid secretion and gastric motility [78], and decreased gastric mucus secretion [82]. As shown in the pre-treatment with Zn (II) complex, there was the same expression pattern (with a direct relation) between the level of secretion of gastric mucosa and the level of PGE-2 in the homogenate [83]. On the other hand, the inhibition percentage was almost in the same pattern with the level of GWM. However, the protection was not appeared in a clear dose-dependent manner. This finding could be due to the possible anti-inflammatory effect of the complex, where the pre-treatment in lower concentrations appeared more effective (with relatively higher inhibition percentage, PGE2 and GWM secretion). Increasing the pre-treatment dose showed more anti-inflammatory effects, astonishingly. Several studies showed that Schiff base derivative compounds possessed anti-inflammatory activity [84]–[86]. The endogenous prostaglandins that contribute to ulcer healing/protection are derived from COX-2 [87]. Some of the Schiff base complexes are selectively COX-2 inhibitors in relatively high concentrations [88], [89] (For a review, see [87]). However, another study should be performed to evaluate the anti-inflammatory effect of the Zn (II) complex and to highlight the exact anti-inflammatory mechanisms in different doses.

Immunohistochemistry evaluation of the gastric tissue for each group confirmed the gastroprotection effect of the pre-treatment, either with the omeprazole (5.790×10^−5^ M/kg) or the zinc (II) complex. Heat shock proteins is classified into four families (HSP90, HSP70, HSP60, and Hsp70). The low molecular weight chaperone, Hsp70 mediates a variety of post translational modification of polypeptides [90]. Many studies have shown the importance of Hsp70 as a cytoprotective protein under various stress conditions [91]–[93]. In consistence with the previous studies [25], [30], [34], the present study demonstrated that the mucosal expression of Hsp70 in those rats pre-treated either with the omeprazole (5.790×10**^−^** ^5^ M/kg) or with the zinc (II) complex was increased when compared with the lesion control group. In the process of gastroprotection, balance between apoptosis and cell proliferation should be maintain. Bcl-2 family consists of different proteins such as Bax and Bcl-2 [94]. Bax protein promotes apoptosis but Bcl-2 protein is an antagonist to the function of Bax [95]. Immunohistochemistry evaluation for Bax protein in the gastric tissue of each group showed that Bax protein was at its highest level of expression in the pre-treatment with ethanol but significantly reduced when the rats pre-treated with omeprazole or the complex. Previous study demonstrated that a copper (II) complex was able to reduce the expression of Bax protein, significantly [25]. A newly published research showed effectiveness of a new Schiff base derived copper (II) complex on gastroprevention [25]. The complex showed the inhibition percentage of that complex in a dose-dependent manner, in which the protection with 80 mg/kg of the complex was the most effective dose. In comparison, this study showed a remarkable protection in lower administrated doses (2.181×10**^−^** ^5^ and 4.362×10**^−^** ^5^ M/kg). The effectiveness of the zinc (II) complex appeared similar to omeprazole (5.790×10**^−^** ^5^ M/kg) but it could make the prevention in significantly lower concentration in comparison to the copper (II) complex.

## Conclusions

The zinc (II){Dichlorido-2-morpholino-*N*-[1-(2-pyridyl)ethylidene] ethanamine *k^3^ N,N’,N”}* complex did not appear toxic in administrated doses (43.621×10**^−^** ^5^ or 87.241×10**^−^** ^5^ M/kg) in mice. The complex could significantly enhance the protective mechanisms of mucosa against acute hemorrhagic mucosal lesions. Antioxidant activities (NO, CAT, SOD and GSH) improved the protection against free radicals and maintain the level of the MDA. The zinc (II) complex, in some extent, stimulated the release of PGE-2 in the gastric tissue homogenates similar to that of omeprazole. The macroscopic and microscopic evaluations of the gastric tissues confirmed the gastroprotective effect of the complex through reduction of epithelial mucosal lesion, submucosal edema and neutrophil infiltration and through increase in glycoprotein content of the gastric homogenate and Hsp70 protein. This study introduced the complex as an efficient gastroprotective agent against acute hemorrhagic gastric lesions in rats.

## Supporting Information

Figure S1 **1H-NMR spectrum.** DMSO-D6 record of the zinc (II) complex [38].
(TIF)

Figure S2 **13C-NMR spectrum.** DMSO-D6 record of the zinc (II) complex [38].
(TIF)

Figure S3 **Microscopic evaluation for the acute toxicity test.** H&E staining for liver (A) and kidney (B) do not show any sign of toxicity in rats received 87.241×10^−5^ M/kg of the complex. There is no significant difference in structures of liver and kidney among the groups.
(TIF)

Table S1 **Acute toxicity test.**
(DOCX)
